The article "Protective Effects of A. sativa against Oxidative Stress-Induced Liver Damage in Ovariectomized Mice" was published in 2021. Journal: Biomed Res Int.

# Protective Effects of *A. sativa* against Oxidative Stress-Induced Liver Damage in Ovariectomized Mice

**DOI:** 10.1155/2021/5577498

**Published:** 2021-07-15

**Authors:** Mabrouka Ltaif, Manel Gargouri, Ahlem Soussi

**Affiliations:** Laboratory of Animal Ecophysiology, Faculty of Sciences, Sfax University, Tunisia

## Abstract

Postmenopausal women express great failure in their ovarian hormone production, especially estrogen. This deficiency may promote hypercholesterolemia and accelerate the redox imbalance. The present study was designed to evaluate the protective effect of *Avena sativa* against estrogen deficiency-induced liver and uterus oxidative injury in experimental ovariectomized mice. Female mice were randomly divided into five groups: group one (negative control) received normal diet and distilled water (C), group two (positive control) received daily enriched diet with oat grains and was kept on tap distilled water at a dose of 200 mg kg^−1^ d^−1^ (A), group three (ovariectomized mice) was nontreated fed with normal diet (O), group four includes ovariectomized mice treated daily with estradiol given by intraperitoneal injection at a dose of 100 *μ*g kg^−1^ d^−1^ (OE), and the fifth group also includes ovariectomized mice which received enriched diet with oat grain parts with the same dose given to group two. The treatment period lasted two consecutive months. Both oat and hormonal treatments of ovariectomized groups resulted in a significant reduction in triglycerides and total cholesterol and increased high-density lipoprotein (HDL) levels in the plasma after 21 and 60 days of treatment. Besides, the coadministration of *A. sativa* has decreased the activities of alkaline phosphatase (ALP) and lactate dehydrogenase (LDH) and increased transaminase activities after 21 and 60 days of treatment. On the other hand, this cereal has restored the enzymatic (SOD, CAT, and GPx) and nonenzymatic antioxidant activities (GSH) as well as the elevated thiobarbituric acid reactive substances (AOPP and PCO) to near-normal values. The beneficial effects of this cereal were confirmed by a histological study of the liver and uterus of all previous cited groups. Our finding emphasized the antioxidant and antilipidemic effect of oat grain part, suggesting the use of this cereal in the prevention of liver and uterus diseases that occurred in postmenopausal women.

## 1. Introduction

It has been demonstrated that menopause is a natural state of ovarian hormone deficiency, defined as twelve consecutive months of amenorrhea. This transition in women's life is probably associated with imbalance between oxidant and antioxidant activities, leading to oxidative cell damage [1, 2].

This imbalance is induced by the overproduction of reactive oxygen species (ROS), highly reactive molecules, generated during cell metabolism. They have deleterious effects on cellular components (proteins, lipids, and DNA), accelerate the aging process, and induce several diseases, such as hyperlipidemia, inflammation, cardiovascular disease, cancer, and arteriosclerosis [3, 4].

The structure and function of different organs are directly influenced by oxidative stress including the liver which is mainly affected. Many investigators have confirmed that menopause is associated with increased risk of dyslipidemia that includes elevated triglycerides, total cholesterol, and lowered high-density lipoprotein (HDL) concentrations in plasma [5, 6].

On that account, liver dysfunction, in postmenopausal women, is strongly related to plasma dyslipidemia and triglyceride accumulation that can also lead to arteriosclerosis and cardiovascular disease [7]. Moreover, epidemiological studies have shown that hepatic steatosis is less common in middle-aged women than in men and have proved that administration of 17*β*-estradiol to ovariectomized mice reduces this steatosis [8, 9]. Thus, we hypothesized that endogenous estrogens have a protective role against hepatic disease and oxidative damage.

Menopausal hormone therapy (MHT) can resolve in part the metabolic disturbances related to estrogen deficiency. However, its prolonged use may be accompanied with high risk of endometrial, uterine, and breast cancer [10, 11].

Therefore, there is a great need to find a natural treatment that has less undesirable side effects and that may reduce the need for currently used drugs. Many experimental studies have mentioned the beneficial effects of diet rich in phytoestrogens having protective effects against postmenopausal diseases [12]. These molecules, identified in many cereals, are known by their estrogenic effect thanks to their similarity with 17*β*-estradiol. They are able to scavenge free radicals and modulate the expression of genes coding for antioxidant enzymes [13]. Many studies on ovariectomized animal models have associated the use of phytoestrogens with a favorable lipid profile [14, 15]. Therefore, plant-derived phytoestrogens are considered to be used as an alternative remedy for the prevention of liver disease in postmenopausal women.

*Avena sativa* is a medicinal plant in the Poaceae family which has been traditionally used for treatment of nervous disorders, rheumatism, and inflammation [16, 17]. In previous studies, it was found that the grain of *A. sativa* had anti-inflammatory and antioxidant effect due to its content in fiber, antioxidants, vitamins, and minerals [18, 19]. In fact, this cereal, known for its richness in manganese, copper, and selenium, acts as a cofactor of several enzymes and participates in the prevention of damage caused by free radicals [20].

In the present study, we report the first in vivo experimental study on the effects of *A. sativa* on liver injury in ovariectomized mice. In vivo and in vitro studies suggested that *A. sativa* clearly prevented hepatic and uteric oxidative damage induced by estrogen deficiency. *A. sativa* modulated the lipid profile, liver and uterus enzyme levels, and antioxidant status of these two organs. Therefore, it could be a potential alternative treatment to prevent postmenopausal hepatic and uteric dysfunction.

## 2. Materials and Methods

### 2.1. Chemical Reagents

NBT (nitro blue tetrazolium chloride), butylated hydroxytoluene (BHT), GSH (reduced form), and all other chemicals used in biochemical assays were purchased from Sigma-Aldrich (Saint Louis, Missouri, USA).

### 2.2. Plants

The grains of *Avena sativa* (Ref: HEMA001004) were purchased from the local pharmacy of Mohamed Dammak in Sfax, Tunisia. To evaluate the antioxidant power of this cereal, an ethanolic extract was prepared by dissolving 2.5 mg of cereal powder in 10 ml of ethanol 95%. Then, this solution was diluted in order to prepare a series of different concentrations from 0 to 0.25 mg/ml.

### 2.3. In Vitro Assays

#### 2.3.1. *β*-Carotene Bleaching Test

The ability of ethanolic oat extract to inhibit *β-*carotene bleaching was evaluated according to the method of Koleva et al. with slight modifications [21]. The absorbance was measured at 470 nm before and after 120 min of incubation at 50°C. Results were expressed as IC_50_ values in mg ml^−1^ calculated using the following formula:

(1) $$\begin{array}{c} \beta ‐\text{carotene bleaching inhibition}\left(\%\right)=\left[\frac{\left(S-C_{120}\right)}{C_{0}-C_{120}}\right]*100, \end{array}$$

where *C*_0_ and *C*_120_ are the absorbance of the control at 0 and 120 min, respectively, and *S* is the sample absorbance at 120 min. The IC_50_ value (mg/l) corresponds to the effective concentration of the sample at which the *β-*carotene bleaching was 50% inhibited.

#### 2.3.2. Superoxide Radical-Scavenging Activity

The superoxide radical scavenging activity was determined according to the method of Martinez et al. [22]. 100 *μ*l of the oat extract, at different concentrations, was mixed with potassium phosphate buffer (67 mM), EDTA (6.45 mM), NBT (0.096 mM), and riboflavin (3.87∗10^−3^ mM) and then exposed for 10 minutes to intense light. Their absorbance was measured at 560 nm, and the superoxide radical-scavenging rate was expressed in IC_50_ (mg/ml) and evaluated according to the following formula:

(2) $$\begin{array}{c} \text{Scavenging rate}\left(\%\right)=\frac{\left(A_{0}-A_{1}\right)}{A_{0}}\times 100, \end{array}$$

where *A*_0_ was the absorbance of the blank and *A*_1_ was the absorbance of the ethanol extract of oats.

#### 2.3.3. Nitric Oxide Scavenging Activity

This essay was determined according to the method of Marcocci et al. [23]. Briefly, the reaction mixture (5 ml) contains sodium nitroprusside in a buffered phosphate solution (0.5 mM, pH = 7.4), with or without ethanolic oat extract at different concentrations. The mixture was incubated at 25°C for 150 minutes in front of a visible polychromatic light source. Then, 0.5 ml of the incubation mixture was mixed with 1 ml of sulfanilamide (1% in 5% phosphoric acid) and incubated at 25°C for 5 minutes. The absorbance was read at 546 nm after a third incubation with 1 ml of 1-naphthyl-ethylenediamine for 30 min at 25°C. The nitric oxide scavenging rate was expressed as IC_50_ values in mg ml^−1^ and calculated using the following formula:

(3) $$\begin{array}{c} \text{Scavenging rate}\left(\%\right)=\frac{\left(A_{0}-A_{1}\right)}{A_{0}}*100, \end{array}$$

where *A*_0_ was the absorbance of the blank and *A*_1_ was the absorbance of the ethanol extract of oats.

#### 2.3.4. Phenolic Compound Determination by HPLC-DAD

The identification of phenolic compounds in the grain of *A. sativa* was done using the HPLC system (consisting of a vacuum degasser, an autosampler, and a binary pump with a maximum pressure of 400 bar; Agilent 1260, Agilent Technologies, Germany) equipped with a reversed-phase C18 analytical column of 4.6 × 100 mm and 3.5 *μ*m particle size (Zorbax Eclipse XDB C18). The DAD detector was set to a scanning range of 200-400 nm. Column temperature was maintained at 25°C. The injected sample volume was 2 *μ*l, and the flow rate of mobile phase was 0.4 ml/min (mobile phase B consisted of 0.1% formic acid and mobile phase A was methanol). The optimized gradient elution was illustrated as follows: 0-5 min, 10-20% A; 5-10 min, 20-30% A; 10-15 min, 30-50% A; 15-20 min, 50-70% A; 20-25 min, 70-90% A; 25-30 min, 90-50% A; and 30-35 min, return to initial conditions. Identification analysis was done by comparison of their retention time with those obtained from the extract. For the quantitative analysis, a calibration curve was obtained by plotting the peak area against different concentrations for each identified compound at 280 nm [24].

### 2.4. *In Vivo* Assays

#### 2.4.1. Animal Treatments and Experimental Design

This study was carried out on 30 Swiss female mice (aged 7-8 weeks), obtained from the Central Pharmacy of Tunis (SIPHAT). They were housed in cages in a breeding farm under controlled laboratory conditions (22 ± 2°C, relative humidity 40 ± 4%, and a 12 h light/dark cycle) with free access to drinking water and diet. The pelleted diet was 22% protein and supplied by the Industrial Company of Concentrate (ALMASS-Sfax, Tunisia).

Experimental protocols were approved by the Ethical Committee of the Faculty of Science of Sfax, protocol number 94-1939, and they were carried out according to the general guidelines on the use of living animals in scientific investigations (Council of European Communities 1986). After two weeks of acclimatization, we removed the two ovaries of the mice belonging to the ovariectomized groups. This operation was performed under general anesthesia after ligation of the vascular pedicles to prevent blood bleeding.

Two weeks postsurgery, we divided the mice into 5 groups as follows.

Group C: negative control group that received distilled water and a normal diet.

Group O: ovariectomized group that received distilled water and normal diet.

Group OE: ovariectomized mice given distilled water and normal diet and administered orally with estrogen at a dose of 100 *μ*g/kg/day^25^.

Group OA: ovariectomized mice received distilled water and fed with a diet enriched with oats grains at a dose of 200 mg/kg/day^26^.

Group A: positive control group that received distilled water and oat-enriched diet with the same dose given to group OA.

After 21 and 60 days of treatment, mice were sacrificed by rapid decapitation. Blood samples were collected in heparinized tubes and centrifuged (3000 g for 15 min). Then, plasma was recovered and stored at -80°C until analysis. The uterus and livers were excised and cleaned. Some samples were homogenized in phosphate buffer solution (pH = 7.4) and centrifuged, and their supernatants were stored at -80°C for biochemical assays. Other uterus and liver samples, immediately removed, were cleaned and fixed in Bouin's solution for histological studies.

#### 2.4.2. Enzyme Kits

Levels of total cholesterol, HDL, aspartate aminotransferase (AST), alanine aminotransferase (ALT), lactate dehydrogenase (LDH), and alkaline phosphatase (ALP) activities in plasma were assayed using commercial reagents kit (Biomaghreb, Tunisia; Ref: 304706, 304342, 304410, 304663, 20012, and 20114, respectively).

#### 2.4.3. Lipase Inhibition Assay

The Lipase Activity Assay Kit (Ref 95801, Biolabo, France) was used to determine lipase activity. According to the operating instructions, 2 mg of oat powder solubilized in 200 *μ*l of mouse serum was combined with lipase in working solution and the final absorbance was read at 550 nm.

#### 2.4.4. Protein Quantification

Liver protein contents were calculated according to the method of Lowry et al. using bovine serum albumin as standard [25].

#### 2.4.5. Estimation of Lipid Peroxidation Levels in the Liver

The level of lipid peroxidation in liver tissues was measured as the amount of thiobarbituric acid reactive substances (TBARS) according to Yagi [26]. Briefly, 125 ml of supernatants was mixed with equal volume of TCA-BHT in order to discard proteins. After centrifugation (1000 g, 10 min, 4°C), 200 ml of the resulting supernatant was mixed with 40 ml of HCl (0.6 M) and 160 ml of thiobarbituric acid (TBA) 20% dissolved in Tris. The mixture was heated at 80°C for 10 min, and after cooling at room temperature, the absorbance was read at 530 nm and TBARS values were calculated and expressed in nmol/mg protein.

#### 2.4.6. Estimation of Advanced Oxidation Protein Products and Protein Carbonyl in the Liver

Advanced oxidation protein product (AOPP) levels in the liver tissue were estimated according to the method of Kayali et al. [27]. The absorbance of the sample was measured at 340 nm, and the concentration of AOPP was calculated using the extinction coefficient of 261 cm^−1^ mM^−1^. The result was expressed as nmol/mg protein.

The protein carbonyl (PCO) content of liver tissue was measured using the method described by Reznick and Packer [28] based on the reaction of the carbonyl groups with 2,4-dinitrophenylhydrazine (DNPH) to form 2,4-dinitrophenylhydrazone. The absorbance of the sample was read at 370 nm, and the carbonyl content was calculated using the molar absorption coefficient for aliphatic hydrazones (22,000 M^−1^ cm^−1^) and expressed as nmol/mg protein.

#### 2.4.7. Enzymatic and Nonenzymatic Status in the Uterus and Liver

Superoxide dismutase (SOD) activity was determined according to the methods of Asada et al. based on the photoreduction of nitro blue tetrazolium (NBT) [29]. The absorbance was read at 560 nm, and the SOD activity was expressed as units/mg protein, knowing that one unit of SOD is defined as the amount of enzyme able to inhibit the photoreduction of NBT by 50%.

The catalase (CAT) activity was determined according to the method of Aebi based to the decrease in absorbance related to the degradation of H_2_O_2_ for 1 min at 240 nm [30]. CAT activity was expressed as mmol H_2_O_2_ consumed/min/mg protein.

Glutathione peroxidase (GPx) activity in the liver was determined according to Paglia and Valentine [31]. GPx activity was measured at 412 nm using a spectrophotometer and expressed as nmoles of reduced GSH/mg protein.

Reduced glutathione (GSH) in liver tissues was measured according to the method of Ellman [32] modified by Jollow et al. [33]. Glutathione content was measured at 412 nm after 10 min and expressed in *μ*g/mg of tissue.

#### 2.4.8. Histopathological Examination

After fixation in Bouin's solution, pieces of fixed uterus and liver tissues were embedded into paraffin, sectioned at a thickness of 5 *μ*m, and stained with hematoxylin-eosin for histological studies. Six slices were prepared from the liver collected from each mice belonging to each group. All sections were evaluated semiquantitatively for the degree of uterus and liver injury. The steatohepatitis calculation system was applied to evaluate necrosis, inflammation, and ballooning [34].

#### 2.4.9. Statistical Analysis

Statistical analysis was performed using one-way analysis of variance (ANOVA), followed by the Fisher test for comparison between groups, and the level of statistical significance was set at *p* < 0.05. Post hoc test was required to be used for comparison between two groups. All values were expressed as means followed by standard deviation (SD). Differences were considered significant at different levels (*p* < 0.05, *p* < 0.01, and *p* < 0.001).

## 3. Results

### 3.1. In Vitro Assays

#### 3.1.1. Antioxidant Activity of *Avena sativa*

The antioxidant activity of *Avena sativa* was measured by the ability of this cereal to inhibit the bleaching of *β*-carotene and to scavenge the superoxide anion (O_2_^·–^) radicals and the nitric oxide (NO^·^). In fact, the presence of antioxidants in our extract minimized the extent of *β*-carotene destruction by neutralizing the free radical of linoleate and any other free radical formed in the system (Figure 1). In this assay, *A. sativa* extract exhibited an interesting antioxidant activity (*μ*g/ml) compared to BHT, a well-known natural antioxidant (IC_50_ = 0.13 ± 0.015 mg/ml) (Table 1). On the other hand, the O_2_^·–^ radical scavenging effect is necessary to prevent the formation of hydroxyl radicals OH^·^ and their deleterious effects. The ability of our plant extract to scavenge this radical resulted in a decrease in the absorbance of the blue formazan solution at 560 nm, and the IC_50_ value was 0.23 ± 0.006 mg/ml compared to the standard antioxidant which is ascorbic acid (Table 1).

Finally, our results showed that the ethanol extract of *A. sativa* exhibited strong NO^·^ scavenging activity leading to the reduction of the nitrite concentration in the assay medium. Indeed, the oat extract in sodium nitroprusside (SNP) solution significantly inhibited (*p* < 0.05) the accumulation of nitrite (IC_50_ = 0.02 ± 0.008 mg/ml), a stable oxidation product of NO^·^, liberated from SNP in the reaction medium with time, compared to the standard ascorbic acid (Table 1).

#### 3.1.2. Measurement of Lipase Inhibitory Activity

According to Table 2, *A. sativa* has a cholesterol-lowering effect demonstrated by the decrease in lipase activity of the serum combined with oat (by 60.13%) as compared to the control.

#### 3.1.3. HPLC Characterization of *A. sativa* Extract

Qualitative analysis of phytoconstituents in the methanolic extract of *A. sativa* revealed the presence of phenolic compounds (Figure 2). Ten different phenolics have been identified through the HPLC finger printing such as quercetin (retention time (RT) = 5.98 min; peak 1), catechin (RT = 13.78 min; peak 2), kaempferol (RT = 15.21 min; peak 3), caffeic acid (RT = 17.23 min; peak 4), syringic acid (RT = 17.63 min; peak 5), ferulic acid (RT = 20.27 min; peak 6), rosmarinic acid (RT = 21.78 min; peak 7), naringenin (RT = 24.45 min; peak8), amentoflavone (RT = 26.94 min; peak9), and myrictin (RT = 29.66 min; peak 10) (Table 3).

### 3.2. In Vivo Study

#### 3.2.1. Effect of Ovariectomy on Hepatic Biomarkers and Lipid Profile

As reported in Table 4, ovariectomy induced abnormal liver function as demonstrated by a significant increase in ALP and LDH activities after 21 days by +43.63% and +45.41%, respectively. The increase in LDH activity persists even after 60 days (by 52.28%) while ALP activity has restored the normal value compared to the control. Conversely, the plasma levels of transaminase, alanine aminotransferase (ALT) and aspartate aminotransferase (AST), did not show significant variations after 21 days; however, at the end of treatment, they were significantly lower (-17.98% and -15.2%) in ovariectomized mice than in the controls. The comparison between results of 21 and 60 days revealed a reduction in ALP and LDH level up to -43.60% and -4.45%, respectively. However, for transaminases (AST and ALT), elevations of 15.22% and reduction of -17.97% were observed, respectively, towards the end of the experiment compared with data of the 21 days.

Changes in lipid profiles (Table 5), revealed by a significant increase in total cholesterol (+48.16% and 20.45% after 21 and 60 days of treatment, respectively), were detected in ovariectomized mice. Similarly, a remarkable rise in triglycerides and VLDL cholesterol level was also recorded in the ovariectomized group after 21 days of treatment (+67.20% and +41.34%, respectively) as well as at the end of the experiment (+20.02% and +23.84%, respectively) when compared with controls. However, a remarkable increase in HDL cholesterol levels in the plasma was evident in the ovariectomized group after 21 days of treatment (+50.68%), whereas an appreciable decrease was detected at the end of treatment (+10.57%).

In addition, ovariectomy has significantly decreased the HTR (%) and increased highly the atherogenic index (AI) as compared to normal mice after 21 and 60 days of treatment (-15.96% and -29.74%, respectively). After the administration of synthetic estrogen or *A. sativa* to ovariectomized mice, a considerable amelioration in plasma hepatic markers was observed. Treatment with oat alone had no effect per se in the levels of the previous tested parameters, but it lowered the level of triglycerides with a slight elevation in the ALP level when compared with the control.

#### 3.2.2. Estimation of TBARS, AOPP, PCO, and Enzymatic and Nonenzymatic Antioxidant Levels in Liver Tissues

Figure 3 shows the hepatic peroxidation levels of control and experimental mice. In the ovariectomized mice, TBARS level, an index of lipid peroxidation, showed a highly significant increase by 77.60% and 9.46% after 21 days and 60 days, respectively.

Similar observations could be made concerning the protein oxidation in the liver of ovariectomized mice which increased markedly, reveled by high levels of AOPP and PCO after 60 days (+36.84% and 26.77%, respectively) (Figure 4). Here again, hormonal treatment and the addition of oat allowed lipid peroxidation, advanced protein products, and protein carbonyls to remain close to control value. The oat group showed no noticeable variation in TBARS, AOPP, and PCO levels compared with the control one.

Concerning the effect of oophorectomy on the enzymatic antioxidant, hepatic SOD activity of female adult mice suffered from estrogen deficiency decreased (by −17.90%) after 21 days; however, after 60 days, it has undergone a remarkable elevation (by +16.24%) as compared to control animals (Table 6).

Similar observations could be made concerning CAT activity in the liver of those mice which showed a remarkable decrease (-55.35%) after 21 days and appreciable increase (+21.36%) after 60 days of experiment. A significant recovery in liver SOD and CAT activity was observed in ovariectomized mice treated with oat or receiving synthetic estrogen (Table 6).

Moreover, GPx activity and GSH content showed a highly significant increase (by +44.63% and +16.24%, respectively) after 21 days in the liver of ovariectomized group compared to controls. Nevertheless, after two months of treatment, GPx and GSH did not show any significant variation. Alternatively, treatment of mice with oat or estrogen decreased hepatic GPx and GSH content after 21 days, as compared to ovariectomized mice. Oat supplementation had no effect per se on enzymatic and nonenzymatic antioxidant activities of this vital organ.

#### 3.2.3. Effect of Ovariectomy on Enzymatic and Nonenzymatic Antioxidant Levels in the Uterus

Based on our results given by Table 7 after three weeks of treatment, there was a significant increase in catalase activity (by +48.6%) and a significant decrease in the activity of SOD and GPx and in the level of GSH in the homogenate of the uterus (by -26.65, 50.72, and 28.76%, respectively) in ovariectomized mice compared to controls (Table 7).

These variations were detected also towards the end of the experiment, and a significant increase in the level of SOD and uterine catalase (by +14.63 and 24.5%, respectively) was recorded in the ovariectomized mice as compared to control mice. On the other hand, a significant decrease was recorded in GPx activity and GSH level (by +29.98% and 17.30%, respectively) after 60 days of treatment in ovariectomized mice compared to controls (Table 7).

The use of oat grains or hormonal treatment restored the levels of these antioxidants to normal values. In our study, the administration of oats to nonovariectomized mice did not affect their antioxidant status and did not show any significant variations when compared to controls.

#### 3.2.4. Histopathological Examination

*(1) In the Liver*. Liver histological examination of the control group showed also a normal histoarchitecture including hepatic lobules consisting of a central vein surrounded by radiating hepatocytes (Figures 5(a) and 5(b)). Nevertheless, in ovariectomized (O) mice, liver histoarchitecture showed leucocyte infiltration, fat droplet accumulation, and binucleated hepatocytes (Figures 5(c) and 5(d)). Administration of 17*β*-estradiol in mouse groups improved partially the histological alterations induced by ovariectomy (Figures 5(e) and 5(f)). Contrariwise, the liver had a nearly normal appearance: no leucocyte infiltration but some traces of lipids that remain (Figures 5(g) and 5(h)).

The histopathological scoring reflected the findings from the microscopic observation of the hepatic tissue (Table 8).

*(2) In the Uterus*. After staining with hematoxylin-eosin, 3 layers appeared in the uterus of mice such as the perimetrium, myometrium, and endometrium. Uterus sections of the control mice showed normal perimetrium, myometrium, and endometrium, well-developed endometrial glands, and a distinct vascularization (Figure 6(a′)). Ovariectomy in rats (group O) provoked histological changes in uterus tissue and an atrophied endometrium and myometrium with a compact stroma. Atrophied endometrial glands and a poor vascularity were shown (Figure 6(b′)). Treatment with oats (Figure 6(d′)) showed more significant improvement than hormone treatment (Figure 6(c′)). In the myometrium and endometrium, we detect a moderate hypertrophy in these two layers compared to untreated ovariectomized mice.

The severity of these histomorphological changes was scored and presented in Table 9.

## 4. Discussion

Cereals have a long history of use, and they have reached a new high interest in recent years including therapeutic attention [35]. Among cereals, oat (*Avena sativa*) is distinct by its various components and nutritional profile. It is a good source of dietary fiber, protein, fat, minerals, and vitamins [36, 37]. Most reported investigations focused on specific oat components, such as *β*-glucans, tocopherols (vitamin E), or avenanthramides. However, studies on whole oat grains with respect to antioxidant and antilipidemic activities are still lacking.

Therefore, the antioxidant and antilipidemic power of *A. sativa* application has been studied *in vitro*. The antioxidant potential of the grain ethanolic extracts was assessed on the basis of *β*-carotene bleaching test and superoxide anion and nitric oxide scavenging activity. Our results showed that *A. sativa* extract exhibited a high ability to inhibit *β*-carotene bleaching (IC_50_ = 0.13 ± 0.015 mg/ml) and it was nearly as active as the standard antioxidant, butylated hydroxytoluene (BHT). Interestingly, the ethanolic extract of oat grain parts scavenge strongly the superoxide anion (IC_50_ = 0.23 ± 0.006 mg/ml), highly reactive oxygen species, even better than the standard ascorbic acid. Our results were in agreement with previous finding which highlighted that oat had very important oxygen radical absorption capacity compared with other whole grains [38, 39]. In addition, our extract moderately inhibited nitric oxide radicals with the IC_50_ value being 0.002 mg ml^−1^.

The overproduction of this radical can induce tissue damage and associated with inflammatory diseases such as atherosclerosis and hypertension [40]. These data are related to the content in phenolic compounds, responsible to the inhibitory effect of oat ethanolic extract.

These molecules were identified using the HPLC method. According to the retention time of calibration standards, oat methanolic extract showed a chemical profile composed of ten identified phenolic compounds, including quercetin, catechin, kaempferol, caffeic acid, syringic acid, myrictin, rosmarinic acid, naringenin, amentoflavone, and ferulic acid. The presence of these compounds in oat extracts approved the interesting biological activity of this cereal. In fact, previous studies showed that these phenolic compounds are potent scavengers of free radicals and are potentially useful in the prevention of many diseases such as arteriosclerosis, diabetes, and cancers [41]. Results showed that the major compounds in *A. sativa* were ferulic acid, rosmarinic acid, amentoflavone, and myrictin. Ferulic acid is a high-potency phenolic compound, beneficial in the treatment of various disorders linked to oxidative stress, such as aging skin, diabetes, and neurodegenerative disease [42]. Besides, it has been shown to play a vital role in providing the rigidity of the cell wall and have wide biological activity such as anti-inflammatory, antimicrobial, antithrombotic, hepatoprotective, and vasodilator action [43, 44]. In addition, rosmarinic acid is a polyphenol similar to caffeic acid. It has also been reported to have anti-inflammatory, antioxidant, and antiviral activities and protect against neurodegenerative diseases [45]. Moreover, amentoflavone and myrictin are interesting flavonoids known by their powerful antioxidant and free radical-scavenging activities and may improve lipid profile by inhibition of LDL oxidation and minimizing the uptake of oxidized LDL by macrophages [46]. These properties can explain its high ability to inhibit lipase activity in the working solution which highlighted its antihypercholesterolemic effect demonstrated by recent researchers [47, 48].

Antioxidant and antilipidemic properties were then analyzed in vivo on ovariectomized female mouse model. It is well known that postmenopausal women who have a decrease in the concentration of estrogen in circulation express disorders in the function of many vital organs such as uterine and hepatic tissue [49]. In fact, this later is the most important metabolic site where a great part of carbohydrate, protein, and lipid metabolism is accomplished [50]. These functions involve several enzymes such as transaminase, ALP, and LDH, and their regulation is carried out by interactions of several factors among which we note the steroid hormones specifically estrogen [51, 52]. In fact, middle-aged women are found to be protected from the risk of developing hepatic diseases when compared to men of similar age [53]. Nevertheless, the change in sex steroidal hormonal profile, after menopause, minimizes this protection. Furthermore, several bibliographic data has demonstrated that bilateral removal of the ovaries is a surgical procedure widely used for induction of liver dysfunction in experimental animals [54].

In this study, ovariectomy was found to cause liver cell damage revealed by several hepatic enzymes including ALT, AST, ALP, and LDH. They are important biomarkers widely used to evaluate the hepatic disorders [55]. Aminotransferases (AST, ALT) are commonly analyzed in serum to assess the possible liver infections and damage. Our findings showed a significant decrease in both AST and ALT activity in ovariectomized mice after 60 days of treatment. Our results were in agreement with previous studies in which plasmatic transaminase levels were declined as indicator of hepatocyte membrane damage [56]. The same results were found by Dong et al. who attributed this significant decrease to the loss of functional integrity of hepatic cell membrane [57]. Therefore, its cells spill out the enzymes like LDH and ALP into the blood. Our data showed also that LDH activity increased in the plasma after 21 days of surgery confirming again the damage in hepatocellular membrane leading to the leakage of this intracellular enzyme into the extracellular fluid. Our results are in agreement with previous investigations reported the elevated activity of this enzyme in the plasma of nontreated ovariectomy mice [58]. Likewise, ALP is found in the majority of tissues and very largely involved in bone metabolism as well as in liver function. Their dosage makes it possible to detect various pathologies especially in the liver [59]. Our finding showed that ALP activity exhibited significant increase at 21 days and restored normal values at 60 days of treatment.

Interestingly, after treatment with oat grain or with estradiol, variation in levels of plasma enzymes (AST, ALT, ALP, and LDH) was totally reduced. In addition to liver enzymes, other lipid parameters may influence liver function such as cholesterol and triglycerides. They are fatty substances that our body needs, at low doses, to build its cells and certain hormones.

However, the excess of these lipids with age contributed to dyslipidemia and increases the risk of onset of liver diseases [60, 61]. In our study, ovariectomy was found to cause concomitant decrease in HDL cholesterol and high elevation in TG and total cholesterol after 21 and 60 days of the surgery. These changes in lipid profile could be related to the estrogen deficiency after the removal of both ovaries. In fact, this hormone has a direct action in lipid metabolism by activating genes required for the uptake and *β*-oxidation of fatty acids and to reduce the expression of genes coding for enzymes used for lipid synthesis such as acetyl-CoA carboxylase 1 (ACC-1) and fatty acid synthase (FAS) [62]. Consequently, with postmenopausal estrogen deficiency, lipid metabolism will likely expect to divert from fatty acid oxidation to fatty acid biosynthesis and TG accumulation [63]. In this study, oat treatment significantly reduced the elevated levels of TG and total cholesterol which confirms its lipid-lowering effect. Likewise, oat supplementation not only lowered T-Ch and TG but also increased HDL cholesterol having the role of transporting cholesterol from the body tissues to the liver, where it will be degraded and recycled. The same results were found by using the hormonal treatment.

Alternatively, it has been reported that ovariectomy can be associated with excessive ROS production responsible for the alterations in membrane structure and function of the liver and uterus, leading to lipid peroxidation as well as protein oxidation [64, 65]. Data from the current study revealed that ovarian dysfunction resulted in an enhanced lipid peroxidation, as indicated by a significant increase of TBARS levels in the liver and uterus tissue as well as a significant increase in protein oxidation, reveled by high levels of AOPP and PCO production. Our data were in agreement with previous research showing that estrogen deficiency develops oxidative damage and metabolic alterations in several organs, including the liver and uterus [66–68].

These finding confirmed the oxidant effect of estrogen deprivation which leads to the alteration of membrane integrity and proteins in cells [69]. Furthermore, this steroid is known by its antioxidant properties; hence, failure in its production results in oxidative stress generation [70].

Furthermore, steroid hormones play an importing role in controlling metabolism and development of several body organs; hence, their absence in the circulating blood may explain the alteration of the enzymatic and nonenzymatic defense system in the liver and uterus of the experimental postmenopausal model used in our study [71]. After 21 days of treatment, activities of SOD and CAT were decreased in the liver of ovariectomized mice, reflecting a response towards free radical damage. In agreement with our findings, the same observations were illustrated by Rodrigues et al. [72]. For the uterus, after three weeks of oophorectomy, there was a decrease in SOD enzymatic activity and an increase in catalase activity. These results can be related to the irreversible inactivation of H_2_O_2_ molecule which leads to the decrease of SOD activity, while CAT activity increased to eliminate these toxic substances [73]. Indeed, the imbalance between the activities of these two enzymes could be explained by the increase of SOD mRNA expression and the inhibition of CAT activity by the superoxide [74].

The increase of their activity after 60 days of treatment, in uterus and liver tissues, can be explained as a response of the body to eliminate accumulated molecules of superoxide anion and hydrogen peroxide [75]. GPx activity and GSH liver content exhibited important increase at 21 days and restored normal value at the end of experiment which can be related to the neutralization of most free radicals generated at the beginning of treatment and the installation of the prooxidant-oxidant balance [76]. Our findings were in accordance with Hamden et al. who have demonstrated that low estrogen levels are responsible for enhanced-free radical generation leading to disruption of the antioxidant status in the liver [13]. The decrease in GPx activity and GSH detected in uterus tissue at 21 days and at the end of treatment demonstrates the alteration of the antioxidant status in this organ [77].

Oxidative damage was confirmed by histological studies which showed mainly a decrease in the thickness of the endometrium and myometrium of the uterus and fat droplet accumulation in liver tissues. Structural alterations of the uterus were confirmed by Danilovich et al. and described a decrease in stroma and glandular epithelium depth observed in the uterus of infertile mice [78]. Several other studies have also confirmed this histological modification in the hepatocytes of ovariectomized animals [79, 80].

The findings from the present study revealed that *Avena sativa* ameliorated significantly the lipid profile, the leakage of hepatic enzymes, and the antioxidant status in hepatic cells of ovariectomized mice. These results are strongly related to its antilipidemic and antioxidant power that allows them to revert dyslipidemia and hepatic oxidative stress associated with estrogen deficiency.

Interestingly, oat treatment significantly reduces the imbalance between ROS generation and scavenging enzyme activities observed in ovariectomized mice. Their protective effect may be related with its phenolic components, detected through the HPLC method. This phytochemical analysis allowed us to confirm its richness in term of phenolics, responsible to their antioxidant power. Besides, the presence of a phytoestrogenic substance, kaempferol, with a structure similar to estradiol, can bind and subsequently activate specific estrogen receptors such as the antioxidant defense gene [81]. Likewise, previous data reported that the molecule of naringenin, detected in our fraction, has an estrogenic activity by interactions with estrogen receptors [82]. Added to that, similar studies have shown that polyphenols in oats have a high cytoprotective activity related to their widely known antiradical property, especially iron-chelating effectiveness [83, 84]. Furthermore, flavonoids in our cereal are well known to possess multiple biological activities including antioxidant, hepatoprotective, antiviral, anticarcinogenic, and vasodilatory actions [85].

## 5. Conclusion

In summary, our hypothesis that *Avena sativa* supplementation could protect mouse liver and uterus against estrogen deficiency-induced changes in lipid profile, levels of hepatic biomarkers, and antioxidant status was accepted. In addition, the results obtained by the use of this cereal were close to those given by the hormonal treatment.

Potent-free radical scavenging, antilipidemic effect, phenolic components, lipid peroxidation, and protein oxidation inhibition of oat grain have been highlighted and can clearly explain the observed hepatoprotective effect of *Avena sativa*. Therefore, the present study provides the biological evidence supporting the use of oat against hyperlipidemia-induced steatosis in liver tissue and perturbations in the uterus confirmed by the histopathological study.

## Figures and Tables

**Figure 1:** Antioxidant power of the ethanol extract of *A. sativa* evaluated by the method of bleaching of *β*-carotene. Each value represents the mean of three trials ± SD.

**Figure 2:** HPLC-MS chromatogram profile of (a) standard and (b) methanolic extract of *Avena sativa* (a: quercetin; b: catechin; c: kaempferol; d: caffeic acid; e: syringic acid; f: ferulic acid; g: rosmarinic acid; h: naringenin; i: amentoflavone; j: myrictin).

**Figure 3:** Lipid peroxidation levels (TBARS) in the liver of controls and treated ovariectomized mice during 21 and 60 days. Values are expressed as means ± SD of 6 mice per group. One-way ANOVA followed by Fisher's protected least significant difference test as a post hoc test for comparison between groups. Comparison between the O or A or OA or OE group and the control (C) group: ^∗^*p* < 0.05; ^∗∗^*p* < 0.01; ^∗∗∗^*p* < .001. Comparison between the OE or OA group and the ovariectomized (O) group: *^+^p* < 0.05; ^++^*p* < 0.01; ^+++^*p* < 0.001.

**Figure 4:** Advanced oxidation protein product (AOPP) and protein carbonyl (PCO) levels in the liver of controls and treated ovariectomized mice in 60 days. Values are expressed as means ± SD of 6 mice per group. One-way ANOVA followed by Fisher's protected least significant difference test as a post hoc test for comparison between groups. Comparison between the O or A or OA or OE group and the control (C) group: ^∗^*p* < 0.05; ^∗∗^*p* < 0.01; ^∗∗∗^*p* < 0.001. Comparison between the OE or OA group and the ovariectomized (O) group: ^+^*p* < 0.05; ^++^*p* < 0.01; ^+++^*p* < 0.001.

**Figure 5:** Photomicrograph of the liver stained with hematoxylin-eosin after (a, c, e, g) 21 days and (b, d, f, h) 60 days of treatment (magnification: 200x and 400x). (a, b) The control group showing normal histoarchitecture including hepatic lobules consisting of a central vein surrounded by radiating hepatocytes. (c, d) Ovariectomized mice showing leucocyte infiltration, fat droplet accumulation, and binucleated hepatocytes. (e, f) Ovariectomized mice treated with estradiol by gavage showing partially improved histology. (g, h) Ovariectomized mice treated with oat by gavage showing no leucocyte infiltration but a few lipid accumulations remained.

**Figure 6:** Photomicrograph of the uterus stained with hematoxylin-eosin after (a′–d′) 60 days of treatment (magnification: 400x). (a′) The control group showing normal histoarchitecture including the perimetrium (P), myometrium (My), endometrium (End), and lamina propria (Lp). (b′) Ovariectomized mice showing compact stroma and an atrophied perimetrium (P), myometrium (My), and endometrium (End) with small endometrial glands (EG). (c′) Ovariectomized mice treated with estradiol by gavage showing partially improved histology. (d′) Ovariectomized mice treated with oat by gavage showing normal function.

**Table 1:** Antioxidant activities of the ethanolic extract of *A. sativa.*

Test	^a^ *β*-Carotene bleaching		^b^(O_2_^·−^)		^c^NO	
Ethanol extract	*Avena sativa*	BHT	*Avena sativa*	Ascorbic acid	*Avena sativa*	Ascorbic acid
IC_50_ (mg/ml)	0.13 ± 0.015	0.11 ± 0.003	0.23 ± 0.006	0.025 ± 0.005	0.02 ± 0.008	0.17 ± 0.006

Values represent the means ± SD of 3 replicates. ^a^*β*-Carotene bleaching (mg ml^−1^). ^b^O_2_^·–^: superoxide anion radical scavenging activity (mg ml^−1^). ^c^NO: nitric oxide scavenging activity (mg ml^−1^).

**Table 2:** Lipase activity (UI) of control serum (C) and serum mixed with oats (C+A).

Groups	Lipase activity
C	0.003 ± 0.0003
C+CA	0.001 ± 0.0002

Values are expressed as means ± SD of 6 assays in each group. One-way ANOVA followed by Fisher's protected least significant difference (FLSD) as a post hoc test for comparison between groups. Comparison between the C+A and control (C) groups: ^∗^*p* < 0.05; ^∗∗^*p* < 0.01; ^∗∗∗^*p* < 0.001.

**Table 3:** Phenolic components separated from oat grain by reversed-phase HPLC.

Phenolic components	Retention time
(1) Quercetin	5.98 min
(2) Catechin	13.78 min
(3) Kaempferol	15.21 min
(4) Caffeic acid	17.23 min
(5) Syringic acid	17.63 min
(6) Ferulic acid	20.27 min
(7) Rosmarinic acid	21.78 min
(8) Naringenin	24.45 min
(9) Amentoflavone	26.94 min
(10) Myrictin	29.66 min

Peaks: (1) quercetin, (2) catechin, (3) kaempferol, (4) caffeic acid, (5) syringic acid, (6) ferulic acid, (7) rosmarinic acid, (8) naringenin, (9) amentoflavone, and (10) myrictin.

**Table 4:** Hepatic biomarkers in the plasma of the control and the ovariectomized mice treated with estrogen or *Avena sativa* for 21 and 60 days.

Treatments	C	A	O	OE	OA
ALP (UI/l)					
21 days	68.00 ± 2.08	74.30 ± 10.9^∗^	97.67 ± 0.67^∗∗∗^	72.66 ± 2.19^++^	64.00 ± 9.40^+^
60 days	92.33 ± 2.73	117.00 ± 1.15^∗∗∗^	90.00 ± 3.00	103.33 ± 6.36	88.00 ± 1.00
LDH (UI/l)					
21 days	1877.66 ± 115.70	1783.50 ± 63.00	2730.00 ± 81.00^∗∗^	2211.25 ± 36.49^∗^^++^	2046.00 ± 77.20^++^
60 days	1824.67 ± 121.62	1652.67 ± 173.67	2571.67 ± 174.18^∗^	2355.67 ± 147.90^∗^	1759.33 ± 275.68
AST (UI/l)					
21 days	361 ± 10.116	330 ± 26.85	376.67 ± 16.33	398.50 ± 56.84	358.50 ± 10.78
60 days	330.23 ± 12.04	284.20 ± 8.16	280.07 ± 10.16^∗^	329.93 ± 13.78^+^	289.73 ± 13.27
ALT (UI/l)					
21 days	45.5 ± 2.598	46.50 ± 5.17	52.00 ± 5.00	49.50 ± 2.933	46.80 ± 3.60
60 days	47.15 ± 1.44	53.83 ± 3.74	38.68 ± 1.82^∗∗∗^	43.43 ± 1.83	42.10 ± 4.14

Values are expressed as means ± SD of 6 mice per group. One-way ANOVA followed by Fisher's protected least significant difference test as a post hoc test for comparison between groups: C: control; A: normal mice fed on *Avena sativa*; O: ovariectomized mice; OE: ovariectomized mice treated with estrogen; OA: ovariectomized mice fed on *Avena sativa*. Comparison between the O or A or OA or OE group versus the control (C) group: ^∗^*p* < 0.05; ^∗∗^*p* < 0.01; ^∗∗∗^*p* < 0.001. Comparison between the OE or OA group and the ovariectomized (O) group: ^+^*p* < 0.05; ^++^*p* < 0.01; ^+++^*p* < 0.001.

**Table 5:** Lipid profile in the plasma of the control and ovariectomized mice treated with estrogen (OM) or with *Avena sativa* for 21 and 60 days.

Treatments	C	A	O	OE	OA
TC (mmol/l)					
21 days	1.80 ± 0.04	1.90 ± 0.264	2.67 ± 0.07^∗∗∗^	2.167 ± 0.133^∗^^+^	1.96 ± 0.120^++^
60 days	2.93 ± 0.06	3.30 ± 0.26	3.53 ± 0.03^∗∗^	6.67 ± 0.012^++^	2.48 ± 0.09^∗^^+++^
TG (mmol/l)					
21 days	1.19 ± 0.03	1.13 ± 0.08	1.98 ± 0.19^∗∗^	1.45 ± 0.03^∗∗^^+^	1.26 ± 0.14^+^
60 days	3.80 ± 0.06	3.267 ± 0.05^∗∗^	4.640 ± 0.12^∗∗^	3.380 ± 0.14^∗^^++^	3.358 ± 0.07^∗∗^^+++^
HDL-Ch (mmol/l)					
21 days	1.65 ± 0.08	1.81 ± 0.18	2.48 ± 0.132^∗∗^	2.06 ± 0.215^∗^	1.94 ± 0.23^+^
60 days	2.60 ± 0.05	3.05 ± 0.31	2.33 ± 0.08^∗∗^	2.37 ± 0.08	2.29 ± 0.05^∗^
VLDL-Ch (mmol/l)					
21 days	0.53 ± 0.003	0.49 ± 0.029^∗∗^	0.90 ± 0.09^∗∗^	0.658 ± 0.019^∗∗^^++^	0.49 ± 0.066^+++^
60 days	1.703 ± 0.013	1.485 ± 0.021^∗∗∗^	2.109 ± 0.064^∗∗^	1.536 ± 0.064^++^	1.526 ± 0.035^∗∗^^+++^
Atherogenic index (AI)					
21 days	0.14 ± 0.031	0.010 ± 0.016	0.26 ± 0.003^∗^	0.094 ± 0.064^+^	0.015 ± 0.017^++^
60 days	0.144 ± 0.010	0.126 ± 0.012	0.555 ± 0.067^∗∗^	0.147 ± 0.003^++^	155 ± 0.003^++^
HRT (%)					
21 days	1.05 ± 0.047	1.03 ± 0.013	0.88 ± 0.03^∗^	0.95 ± 0.043	1.01 ± 0.17^++^
60 days	0.874 ± 0.008	921 ± 0.029	0.614 ± 0.006^∗∗∗^	0.890 ± 0.017^+++^	0.919 ± 0.052^++^

Values are expressed as means ± SD of 6 mice per group. One-way ANOVA followed by Fisher's protected least significant difference test as a post hoc test for comparison between groups. T-Ch: total cholesterol; TG: triglycerides; HDL-Ch: high-density lipoproteins of cholesterol; VLDL-Ch: very low-density lipoprotein-C = TG (mmol/l)/2.2; atherogenic index (AI) = (T‐Ch − HDL‐Ch)/HDL‐Ch; HTR% = HDL‐Ch/T‐Ch ratio. C: control; A: normal mice fed with *Avena sativa*; O: ovariectomized mice; OE: ovariectomized mice treated with estrogen; OA: ovariectomized mice fed with *Avena sativa*. Comparison between the O or A or OA or OE group and the control (C) group: ^∗^*p* < 0.05; ^∗∗^*p* < 0.01; ^∗∗∗^*p* < 0.001. Comparison between the OE or OA group and the ovariectomized (O) group: ^+^*p* < 0.05; ^++^*p* < 0.01; ^+++^*p* < 0.001.

**Table 6:** Antioxidant system activities of controls and ovariectomized treated mice for 21 and 60 days.

Treatments	C	A	O	OE	OA
^a^SOD					
21 days	30.84 ± 0.06	30.20 ± 0.67	22.8 ± 2.6^∗^	25.93 ± 3.08	29.58 ± 1.47^+^
60 days	66.35 ± 2.19	66.44 ± 2.07	77.12 ± 2.65^∗^	68.31 ± 1.29^++^	69.17 ± 1.34^+^
^b^CAT					
21 days	47.19 ± 5.48	44.96 ± 3.89	21.07 ± 2.93^∗∗^	44.22 ± 6.04^+^	40.10 ± 2.07
60 days	48.42 ± 2.38	56.47 ± 0.58^∗^	68.0.6 ± 6.52^∗^	56.70 ± 7.97	56.97 ± 0.03
^c^GPx					
21 days	1.71 ± 0.15	1.72 ± 0.14	2.48 ± 0.17^∗^	2.06 ± 0.10^+^	1.95 ± 0.14^+^
60 days	2.41 ± 0.10	2.55 ± 0.10	2.62 ± 0.05	2.72 ± 0.11	2.67 ± 0.07
^d^GSH					
21 days	0.15 ± 0.02	0.15 ± 0.05	0.17 ± 0.01^∗^	0.15 ± 0.03	0.14 ± 0.02^+^
60 days	0.14 ± 0.03	0.14 ± 0.05	0.15 ± 0.01	0.16 ± 0.04^∗^	0.15 ± 0.04

Values are expressed as means ± SD of 6 mice per group. One-way ANOVA followed by Fisher's protected least significant difference test as a post hoc test for comparison between groups. ^a^SOD: superoxide dismutase (U SOD/mg protein); ^b^CAT: catalase (U/mg protein); ^c^GPx: glutathione peroxidase (nmol/mg protein); ^d^GSH: reduced glutathione (*μ*mol/g tissue weight). C: control; A: normal mice fed with *Avena sativa*; O: ovariectomized mice; OE: ovariectomized mice treated with estrogen; OA: ovariectomized mice fed with *Avena sativa*. Comparison between the O or A or OA or OE group and the control (C) group: ^∗^*p* < 0.05; ^∗∗^*p* < 0.01; ^∗∗∗^*p* < 0.001. Comparison between the OE or OA group and the ovariectomized (O) group: ^+^*p* < 0.05; ^++^*p* < 0.01; ^+++^*p* < 0.001.

**Table 7:** Activities of the uterine antioxidant system of controls and ovariectomized treated mice for 21 and 60 days.

Treatments	C	A	O	OE	OA
^a^SOD					
21 days	10.13 ± 0.68	10.26 ± 0.47	7.43 ± 0.36^∗∗^	10.08 ± 0.36^++^	10.09 ± 0.33^++^
60 days	10.10 ± 0.47	10.02 ± 0.30	11.83 ± 0.45^∗∗^	10.95 ± 0.14^+^	10.95 ± 0.25^+^
^b^CAT					
21 days	4.51 ± 0.64	4.72 ± 0.28	8.70 ± 0.39^∗∗^	6.11 ± 0.42^++^	6.04 ± 0.45^++^
60 days	4.39 ± 0.32	4.54 ± 0.55	5.83 ± 0.17^∗∗^	4.68 ± 0.461^+^	4.97 ± 0.24^+^
^c^GPx					
21 days	6.21 ± 0.41	6.07 ± 0.40	3.06 ± 0.42^∗∗^	6.11 ± 0.22^++^	5.90 ± 0.24^++^
60 days	6.47 ± 0.20	6.29 ± 0.35	4.53 ± 0.30^∗∗^	6.24 ± 0.40^++^	6.37 ± 0.21^++^
^d^GSH					
21 days	0.07 ± 0.002	0.07 ± 0.003	0.05 ± 0.002^∗∗^	0.07 ± 0.002^++^	0.06 ± 0.004^++^
60 days	0.05 ± 0.002	0.06 ± 0.003	0.04 ± 0.001^∗∗^	0.05 ± 0.003^++^	0.05 ± 0.002^++^

Values are expressed as means ± SD of 6 mice per group. One-way ANOVA followed by Fisher's protected least significant difference test as a post hoc test for comparison between groups. ^a^SOD: superoxide dismutase (U SOD/mg protein); ^b^CAT: catalase (U/mg protein); ^c^GPx: glutathione peroxidase (nmol/mg protein); ^d^GSH: reduced glutathione (*μ*mol/g tissue weight). C: control; A: normal mice fed with *Avena sativa*; O: ovariectomized mice; OE: ovariectomized mice treated with estrogen; OA: ovariectomized mice fed with *Avena sativa*. Comparison between the O or A or OA or OE group and the control (C) group: ^∗^*p* < 0.05; ^∗∗^*p* < 0.01; ^∗∗∗^*p* < .001. Comparison between the OE or OA group and the ovariectomized (O) group: ^+^*p* < 0.05; ^++^*p* < 0.01; ^+++^*p* < 0.001.

**Table 8:** Grading of the histopathological changes in the liver tissues of negative controls (C), ovariectomized (O), and ovariectomized mice treated either with 17*β*-estradiol (OE) or with *Avena sativa* (OA) after 21 and 60 days, respectively.

Histological scores	21 days			60 days		
	FDA	BNH	LI	FDA	BNH	LI
C	0	0	0	0	0	0
O	+3	+3	+3	+3	+3	+3
OE	+3	0	+2	+2	0	+1
OA	+1	0	0	0	0	0

FDA: fatty droplet accumulation; BNH: binucleated hepatocytes; LI: leucocyte infiltration. C: control mice; O: ovariectomized mice; OE: ovariectomized mice treated with 17*β*-estradiol; OA: ovariectomized mice treated with *Avena sativa*. Scoring was done as follows: none (0), mild (+1), moderate (+2), and severe (+3).

**Table 9:** Grading of the histopathological changes in the uterus tissues of negative controls (C), ovariectomized (O), and ovariectomized mice treated either with 17*β*-estradiol (OE) or with *Avena sativa* (OA) after 60 days.

Histological scores	60 days					
	P	My	End	Lp	bv	EG
C	0	0	0	0	0	0
O	+3	+3	+3	+3	+3	+3
OE	+1	+1	+2	+1	+1	0
OA	+1	0	0	0	0	0

P: perimetrium; My: myometrium; End: endometrium; Lp: lamina propria; EG: endometrial glands; bv: blood vessels. C: control mice; O: ovariectomized mice; OE: ovariectomized mice treated with 17*β*-estradiol; OA: ovariectomized mice treated with *Avena sativa*. Scoring was done as follows: none (0), mild (+1), moderate (+2), and severe (+3).

## Data Availability

All data used to analyze the findings of this study are included in this manuscript.
